The article "The Combination of Three Natural Compounds Effectively Prevented Lung Carcinogenesis by Optimal Wound Healing" was retracted in 2023. Reasons: duplicated images; overlap with earlier publications; original data or images not available; unreliable data.

# The Combination of Three Natural Compounds Effectively Prevented Lung Carcinogenesis by Optimal Wound Healing

**DOI:** 10.1371/journal.pone.0143438

**Published:** 2015-11-23

**Authors:** Linxin Liu, Hong Li, Zhenzhen Guo, Xiaofang Ma, Ning Cao, Yaqiu Zheng, Shengnan Geng, Yongjian Duan, Guang Han, Gangjun Du

**Affiliations:** 1 Institute of Pharmacy, Pharmacy College of Henan University, Jinming District, Kaifeng, Henan Province 475004, China; 2 Department of Oncology, The first hospital Affiliated to Henan University, Kaifeng, Henan Province 475001, China; Macau University of Science and Technology, MACAO

## Abstract

The tumor stroma has been described as “normal wound healing gone awry”. We explored whether the restoration of a wound healing-like microenvironment may facilitate tumor healing. Firstly, we screened three natural compounds (shikonin, notoginsenoside R1 and aconitine) from wound healing agents and evaluated the efficacies of wound healing microenvironment for limiting single agent-elicited carcinogenesis and two-stage carcinogenesis. The results showed that three compounds used alone could promote wound healing but had unfavorable efficacy to exert wound healing, and that the combination of three compounds made up treatment disadvantage of a single compound in wound healing and led to optimal wound healing. Although individual treatment with these agents may prevent cancer, they were not effective for the treatment of established tumors. However, combination treatment with these three compounds almost completely prevented urethane-induced lung carcinogenesis and reduced tumor burden. Different from previous studies, we found that urethane-induced lung carcinogenesis was associated with lung injury independent of pulmonary inflammation. LPS-induced pulmonary inflammation did not increase lung carcinogenesis, whereas decreased pulmonary inflammation by macrophage depletion promoted lung carcinogenesis. In addition, urethane damaged wound healing in skin excision wound model, reversed lung carcinogenic efficacy by the combination of three compounds was consistent with skin wound healing. Further, the combination of these three agents reduced the number of lung cancer stem cells (CSCs) by inducing cell differentiation, restoration of gap junction intercellular communication (GJIC) and blockade of the epithelial-to-mesenchymal transition (EMT). Our results suggest that restoration of a wound healing microenvironment represents an effective strategy for cancer prevention.

## Introduction

Although conventional anticancer therapies, which consist of surgical resection, radiotherapy and chemotherapy, are effective in the management of many patients, they are ineffective for approximately half of cancer patients [1]. Resistance to conventional anticancer therapies in patients with advanced solid tumors has prompted the need for alternative cancer therapies [2]. Accumulating evidence suggests that cells and factors of the tumor microenvironment decisively contribute to not only the survival of primary neoplastic cells but also to the subsequent key events of neoplastic disease progression, including tumor growth, invasion, and metastasis [3]. Epidemiologically, chronic wound states are well-known risk factors for cancer development [4]. Furthermore, aberrant wound healing with chronic inflammation can reportedly promote malignant transformation [5]. These phenomena have further solidified the view of cancer as “a wound that does not heal” [6]. Studies of the role of aberrant wound healing in cancer pathologies will be important for the discovery of novel therapeutics that can promote wound healing or abrogate carcinogenesis in the tumor microenvironment.

Clearing a wound bed of nonviable tissue is increasingly acknowledged as an important step that may facilitate the healing process for a variety of wound types, particularly chronic wounds [7]. Necrotic tissue in the wound bed will significantly delay and in some cases prevent healing, as it may serve as a reservoir for bacterial growth, contain elevated levels of inflammatory mediators that promote chronic inflammation at the wound site, and impair the cellular migration that is necessary for wound repair [8]. However, the factors that dictate the delicate balance between normal wound repair and aberrant wound healing are yet to be fully elucidated. We hypothesized that appropriate regeneration, sufficient oxygen supply and waste elimination may regulate aberrant wound healing and facilitate tumor elimination. To stringently test this wound healing hypothesis, we screened three natural compounds (shikonin, notoginsenoside R1 and aconitine) from wound healing agents and created an optimal wound healing microenvironment. Specifically, we observed the effects of three compounds on carcinogenesis in mice with lung cancer induced by urethane (ethylcarbamate). We found that wound healing–inducing therapy caused normal cells to lose their malignant transformation potential and improve aberrant wound healing, which may in turn allow for the control of tumorigenesis.

## Materials and Methods

### Reagents

Shikonin, Aconitine and Notoginsenoside R1, 98% or higher purity (HPLC), were purchased from Sigma-Aldrich, Inc. (St. Louis, MO,USA) (S1 Fig). Urethane (ethylcarbamate), lipopolysaccharide (LPS), basic fibroblast growth factor (bFGF), heparin, 12-O-tetradecanoylphorbol-13-acetate (TPA), Clodronate and Evans blue were purchased from Sigma Chemical Co. Bleomycin (BLM) from The antibodies used include: E-cadherin, N-cadherin, Vimentin, Nanog, Oct4, Snail1, CD133, Ki-67, cleaved-caspase 3, connexin 43 and fibronectin were obtained from BD Pharmingen. Horseradish peroxidase (HRP)-conjugated goat anti-mouse IgG polyclonal antibody, Peroxidase substrate DAB (3′, 3′-diaminobenzidine) and AEC (3-amino-9-ethylcarbazole) were from Nichirei Bioscience (Tokyo, Japan). The mouse quantitative ELISA kits (TNF-α, MPO, ROS and 8-OHdG) were obtained from R&D Systems.

### Ethics statement

All animal procedures in this study were approved by the Animal Experimentation Ethics Committee of Henan University, all procedures were performed in strict accordance with the Guide for the Care and Use of Laboratory Animals and the regulation of animal protection committee to minimize the suffering and injury.

### Animals

The female BALB/c mice, 5–7 weeks of age, were obtained from Beijing Weitong Lihua Animal Co. All mice were housed in individual ventilated cages under a 12 h light-dark cycles (lights on 7:00 AM to 7:00 PM). The animals were fed standard rodent chow and water and were maintained under pathogen-free conditions within the institutional animal facility. The animals were monitored daily and euthanized humanely by overdose carbon dioxide at the end of the experiment or the first sign of shortness of breath, reduced locomotion and reduced body weight (greater than 20% total body weight). All surgery was performed under general anesthesia by intraperitoneal injection of 45mg/kg pentobarbital sodium, and all efforts were made to minimize suffering.

### Excision wound model and pharmacological properties of screened compounds

BALB/c mice were intraperitoneally anesthetized with pentobarbital sodium (45 mg⁄ kg), the back hair of the animals was shaved, and a full-thickness excisional wound (approximately 10 mm in diameter) was created on the animal’s dorsum using sharp sterilized scissors. The wounds were kept open, and the mice were housed individually. The gross area of the skin wound was photographed by a digital camera D7000 (Nikon, Japan) every week. The wounds were not sutured or covered and healed by secondary intention. Wound healing was analyzed as a percentage of the original wound area. The wound was considered to be completely closed when the wound area was grossly equal to zero.

To screen wound healing agents, mice were treated with selected natural compounds, including alkaloids, saponins, and naphthoquinones, by oral gavage once daily five days before excisional wound for two weeks. Control mice received vehicle in the same manner (0.5% carboxymethylcellulose in PBS).

Pharmacological properties of screened compounds were examined by TPA- induced ear edema, macrophage phagocytosis and blood perfusion. Briefly, mice were treated with screened compounds (2 mg/kg shikonin, 0.2 mg/kg aconitine and 20 mg/kg Notoginsenoside R1 individually) by oral gavage once daily for ten days. Following the last intragastric administration of compounds, the back blood perfusion of mice was recorded using a Laser Speckle Flowmeter (PeriCam PSI, Sweden). Subsequently, ear edema was induced on the right ear with 20 μL TPA (1.0 mg dissolved in 20 μL acetone) delivered to both the inner and outer surfaces of the ear, the left ear was selected as negative control which received 20 μL acetone. After 3 h, mice received an intraperitoneal injection of 1 mg zymosan in 5 mL normal saline. Next 1 h, mice were euthanzed by overdose carbon dioxide, periotoneal exudates was collected to determine the differential counts based on nuclear morphology using Cytofuge and Wright Giemsa staining. Moreover, 7-mm-diameter ear punch biopsies were individually weighed on an electronic balance, and the edema size was calculated based on the weight difference between both ears.

Forty mice were used in excision wound model and another forty mice were used in measure of pharmacological properties, each group included ten mice. At the end of the experiments, none of mice died or showed signs of distress or discomfort.

### Urethane-induced lung adenocarcinoma model

BALB/c mice were administered freshly prepared urethane to induce lung adenocarcinoma according to our previously published protocol [9]. The mice received an intraperitoneal injection of urethane (600 mg/kg body weight) dissolved in sterile 0.9% NaCl once weekly for 10 weeks. In the first experiment, the mice were treated with the selected compounds (2 mg/kg shikonin, 0.2 mg/kg aconitine and 20 mg/kg Notoginsenoside R1 individually or in combination) suspended in 0.5% carboxymethylcellulose by oral gavage once daily for 22 weeks following the first injection of urethane. In the second experiment, the mice were treated with the selected compounds by oral gavage once daily for 15 weeks following the last injection of urethane. Control mice received vehicle (0.5% carboxymethylcellulose in PBS) by oral gavage. During the studies, the health of the mice was monitored daily, and body weights were measured weekly. At the end of the experiment, under anesthesia with pentobarbital sodium (45mg/kg), the lungs were weighed, filled with fixative overnight, transferred to 70% ethanol for 24 h, and examined using a dissecting microscope to count surface polyps in a blinded fashion. The tumor diameter on the surface of the lung was measured with a digital caliper. Tumor volume was expressed in mm3 and calculated as [l×w^2^] × 0.5, where l and w denote length and width, respectively. After tumors were counted, lung tissues were processed for paraffin embedding and histological or immunohistochemical analysis.

The lung tumor incidence, multiplicity, and tumor load (sum of tumor per lung in average) were determined according to previously established criteria [10].

To observe whether urethane-induced lung carcinogenesis is associated with pulmonary inflammation or lung injury, mice were intratracheally injected 3 times at 3-week intervals with either bleomycin (BLM 200 μg in 50 μL PBS) to induce lung injury or lipopolysaccharide (LPS 20 μg in 50 μL PBS) to induce pulmonary inflammation following the first injection of urethane. To deplete macrophage, liposome-encapsulated clodronate was prepared as described previously [11]. Specifically, 100 μL (1 mg) of clodronate liposome suspension in PBS per mouse was injected intraperitoneally 3 times at 3-week intervals following the first injection of urethane. BALB/c mice were also treated with the compounds according to above protocol following the first injection of urethane.

Next day following the last injection of urethane, five mice each group were euthanzed by overdose carbon dioxide and 10% lung homogenates was performed for assays of ROS and 8-OHdG (lung injury) as well as myeloperoxidase (MPO) and TNFα (pulmonary inflammation) by quantitative sandwich enzyme immunoassay technique according to the manufacturer’s instructions.

To examine interaction between carcinogenesis and wound healing microenvironment, excisional wound (1 cm^2^) was created on the animal’s dorsum of three weeks before the end of experiment.

In this study, each group included twenty-two mice, at the end of the experiment, there were no less than twenty mice in each group. In all experimental procedure, one to two mice each group with clear evidence of myocardial infarction were excluded from the study and humanely euthanzed. The endpoint of the experiment was the first sign of shortness of breath, reduced locomotion and reduced body weight (greater than 20% total body weight) because of lung tumors.

### Histological study

Histological sections (5 μm) were stained with hematoxylin and eosin and analyzed. Proliferative lesions in the lungs were classified as hyperplasia, adenoma or adenocarcinoma based on recommendations published by the Mouse Models of Human Cancers Consortium [12]. Lung pathology scored the lung injury according to previously published criteria [13]: grade 0, normal tissue; grade 1, (<20% of the slide), 2 (20%-50% of the slide) and 3(>50% of the slide). The mean score from all examined fields was calculated as the injury score (IS).

### Immunohistochemical study

Lung histological sections (5 μm) from the paraffin blocks were obtained in silanized slides. The sections were deparaffinized, rehydrated and washed in PBS. Antigen retrieval was performed in 10 mM sodium citrate at pH 6.0 for 20 min using a microwave oven. After blocking with 3% hydrogen peroxide for 10 min, the sections were incubated in 10% fetal bovine serum (FBS) in PBS for 2 h. A blocking solution of 0.1% Triton-X and 0.1% bovine serum albumin supplemented with 2% horse serum was used for the nuclear marker stains. The slides were incubated with primary antibodies in an appropriate blocking buffer overnight at 4°C. Cell proliferation was assessed with a primary monoclonal antibody against Ki-67; cell apoptotic changes were assessed with a primary monoclonal antibody against cleaved-caspase 3; and adenocarcinoma was distinguished using a primary monoclonal antibody against lactate dehydrogenase and TIF-1α. Subsequently, the sections were rinsed with PBS and incubated for 1 h at room temperature with horseradish peroxidase (HRP)-conjugated goat anti-mouse IgG polyclonal antibody. The signal was developed using the peroxidase substrate DAB which generated a brown reaction product. The sections were counterstained with hematoxylin and photographed under a microscope. Each case was scored according to the intensity and area of staining. A combined staining score (intensity + extension) of between 0 and 3 was considered to be low expression, whereas a score between 4 and 6 was considered to be high expression.

### Lung barrier permeability assay

The lung barrier function of the mice was assessed with the Evans blue (EB) dye extra-barrier technique to determine the alveolar epithelium integrity [14]. Thirty minutes prior to sacrifice, 50 mg/kg EB was injected via the tail vein. The mice were subsequently sacrificed, and the lungs were removed to prepare the homogenate. Formamide was added to the homogenate, which was then incubated at 37°C for 24 h and centrifuged at 3,000 rpm for 30 min to obtain the supernatant. Subsequently, the optical density of EB in the supernatant was spectrophotometrically determined at 620 nm and calculated according to the EB standard curve.

### Cell culture

Human alveolar basal epithelial cancer cells A549, human normal bronchial epithelium cells BEAS-2B, Human umbilical vein endothelial cells ECV304 and Mouse fibroblasts L929 were purchased from the Chinese Academy of Sciences. A549 cells were grown in RPMI1640 medium supplemented with 10% (v/v) FBS. BEAS-2B cells and ECV304 cells were cultured in DMEM/F12 medium supplemented with 10% (v/v) FBS. L929 cells were cultured in 4.5 g/l glucose DMEM supplemented with 10% FBS. All cells were grown in a humidified atmosphere containing 5% CO_2_ and 95% air at 37°C. For in vitro experiments, Shikonin, Aconitine and Notoginsenoside R1 were dissolved at a concentration of 50 mM in DMSO as a stock solution (stored at-20°C) and then further diluted in cell culture medium to create working concentrations. The maximum final concentration of DMSO was less than 0.1% for each treatment, and was also used as a control.

### Cell transformation assay

The soft agar-based cell transformation assay was performed in 6-well plates. The plates were pre-coated with 0.5% agar in culture medium containing specified concentrations of compounds based on in vivo serum concentration (shikonin 0.2 μM, aconitine 0.02 μM and Notoginsenoside R1 2 μM alone or in combination). Passage-control A549 cells (5 × 10^3^ cells/well) were mixed with RPMI1640 medium containing 0.5% agar to a final agar concentration of 0.33% and transferred to the top of the bottom agar. Colonies were examined under a light microscope after 2 weeks of culture at 37°C and 5% CO_2_.

A tumor sphere assay was performed in ultralow adherent 6-well plates under serum-free, stem cell-selective conditions as previously described [15]. Briefly, A549 cells (5 × 10^3^ cells/well) were resuspended in 0.8% methylcellulose (MC)-based serum-free RPMI1640 medium supplemented with 20 ng/mL EGF, 20 ng/mL bFGF, 4 mg/mL heparin and specified concentrations of compounds. The cells were further allowed to grow for 14 d, and the numbers of spheres were counted with a microscope. All experiments were repeated in triplicate.

### Cell proliferation

A549 or L929 cells or ECV304 cells (1×10^4^cells/well) were incubated in a 96-well plate overnight at 37°C. Cells were treated with specified concentrations of compounds, each condition was tested in six replicates. During the final 4 h of the 48-h incubation, the supernatants were discarded and 100 μL MTT (0.5 mg/ml) was added to each well. After 4 h, the MTT was discarded and 100 μL of DMSO was added to each well. The absorbance of the samples at 570 nm was determined using a plate reader (Elx-800; Bio-Tek, USA). The results of the cell proliferation assay are presented as a percentage of the control cells. All experiments were repeated in triplicate.

### Cell differentiation assay

A549 cells (1 × 10^4^ cells/well) were incubated in a 6-well plate overnight at 37°C. Cells were treated with specified concentrations of compounds, and the medium was exchanged every 2 d for 8 d. The cells were detached by trypsinization, and cell differentiation was assessed by flow cytometry based on the expression levels of CD133, Nanog, Oct4, E-cadherin, N-cadherin, vimentin and Snail. The data were analyzed to calculate the percentage of the cell population in each group using FlowJo 7.6 software. All experiments were repeated in triplicate.

### Epithelial-to-mesenchymal transition (EMT) and gap junction intercellular communication (GJIC) assays

For the EMT assay, BEAS-2B cells were grown to 70% confluency in a 6-well plate. The cells were then treated with control DMEM/F12, urethane, specified concentrations of compounds for 48 h. The cells were collected, resuspended and analyzed by flow cytometry for the expression levels of E-cadherin, N-cadherin, vimentin and fibronectin using sandwiched antibodies. The geometric mean fluorescence of FITC-conjugated anti-IgG was used to measure protein expression.

The GJIC assay was carried out in 6-well plates using the scrape-loading dye transfer technique [16]. BEAS-2B cells were grown to 80% confluence in a 6-well plate; the cells were then treated with control DMEM/F12, urethane, specified concentrations of compounds for 24 h. After exposure to the target compounds, the cell monolayers were rinsed with PBS, scraped with a surgical steel scalpel blade at low light intensity, and incubated with 1 ml of 1 mg/ml Lucifer Yellow solution for 3 min. The cell monolayers were washed with PBS and fixed with 4% paraformaldehyde. The distance between the designated cut and the dye transfer was measured with an inverted fluorescent microscope. All experiments were repeated in triplicate.

### Western blot analysis

Lung samples from tumor-bearing animals were homogenized and sonicated in RIPA buffer on ice. The lysates were then centrifuged at 12,000 rpm for 15 min at 4°C, and the protein concentration was determined using the Bradford protein assay.

Forty micrograms of protein from tissues was separated on a 12% SDS-PAGE gel and electroblotted onto a polyvinylidene difluoride membrane. The immunoblot was incubated with blocking solution (5% skim milk) at room temperature for 1 h, followed by incubation overnight with a primary antibody against Nanog, Oct4, E-cadherin, N-cadherin, vimentin or connexin 43 at 4°C. The blots were washed and incubated with a 1:1,000 dilution of HRP-conjugated secondary antibody for 1 h at room temperature. After washing, the blots were developed using ECL detection reagent (GE Healthcare) and quantitated by densitometry using Image Quant image analysis system (Storm Optical Scanner). All the experiments were performed independently three times at least.

### Statistical analysis

All data are expressed as the mean ± standard deviation and were analyzed with SPSS 17.0 software. The differences between groups were evaluated using one-way analysis of variance (ANOVA) followed by the Tukey test or Dunnett's test. *P* ≤ 0.05 was considered statistically significant.

## Results

### The screened three compounds promoted wound healing

Cancer is often known as a wound that does not heal. Here, we aimed to determine whether a wound healing microenvironment could prevent the development of cancer. To establish a wound healing microenvironment, we first screened wound healing agents in a skin excision wound model. Among the screened compounds, shikonin, notoginsenoside R1 and aconitine resulted in significantly smaller wound areas during the experimental period than the other compounds (Fig 1A and S1 Table). After 14 d, all wounds treated with shikonin, aconitine and notoginsenoside R1 showed complete closure (10/10), whereas only 50% (5/10) of control wounds showed complete closure. Of note, many hairs were observed in the regenerated skin upon gross evaluation, especially in the aconitine group compared with the other groups.

**Fig 1:** The pharmacological properties of screened three wound healing agents. (A) Screened three compounds promoted wound closure in a skin excision wound model. (B) Notoginsenoside R1 and aconitine increased blood flow perfusion on laser speckle imaging. (C) Shikonin exerted anti-inflammatory efficacy in the TPA-induced ear edema model. (D) Notoginsenoside R1 and aconitine promoted macrophage phagocytosis of zymosan. The results are presented as mean±SE (n = 10/group). ** *p* < 0.01, vs. control group.

In laser speckle imaging, significantly greater blood flow was detected in the wound areas in the notoginsenoside R1 and aconitine groups but not in shikonin group relative to the control group (Fig 1B). Exposing the ears of the mice to TPA to induce edema resulted in marked increases in skin thickness, but this change (the ratio of 2×normal ear thickness and edema ear thickness) was significantly less pronounced in the shikonin group (95.64 ± 5.17%) relative to the TPA control group (82.25 ± 8.92%). Treatment with shikonin reduced the water content in TPA-treated ears by approximately 55% (Fig 1C). The results of the macrophage phagocytosis assay showed that notoginsenoside R1 and aconitine considerably enhanced the macrophage phagocytosis of zymosan in vivo by approximately 25% and 50%, respectively (Fig 1D).

### Histopathology of mouse lung carcinogenesis

To observe the effect of a wound healing-like microenvironment on tumorigenesis, we established a urethane-induced lung carcinogenesis model. In this carcinogenetic model, all mice (20 per group) in the control group developed tumors. During the study, the carcinogenic agents showed slight toxicity without a significant effect on body weight and lethality in less than twenty percent of mice. Most tumors arose centrally within the bronchi at different levels, including the main, lobar, segmental and subsegmental bronchi.

Urethane-induced lung histological alterations were significantly improved by treatment of screened wound healing agents (S2 Fig).

### The combination of three wound healing agents decreased incidence of mouse lung carcinogenesis

To observe the effect of the wound healing microenvironment on lung carcinogenesis, we used three of the screened compounds (shikonin, aconitine and notoginsenoside R1) wich promote wound healing to treat mice following the first or last carcinogen application.

All of the three compounds appeared to prevent carcinogenesis when administered alone following the first carcinogen treatment based on the lung tumor incidence and load, whereas the combination of the three drugs almost completely abrogated urethane-induced lung carcinogenesis based on either lung tumor incidence or load (Fig 2A). However, individual treatment with any of these compounds after the last carcinogen treatment did have no impact on tumor incidence, although the tumor load was decreased (Fig 2B and Fig 3A). Nevertheless, the combination of these three agents remained effective even after the induction of carcinogenesis. As shown in Fig 2C, when the mice were treated following the first carcinogen treatment, the incidences of lung tumorigenesis in the shikonin, aconitine and notoginsenoside R1 groups were 70% (14/20), 50% (10/20) and 65% (13/20), respectively, and these values were significantly lower than that in the control group 100% (20/20). In the combined treatment group, only 10% (2/20) of mice had developed tumors at terminal sacrifice. When the mice were treated following the last carcinogen treatment, the incidence of lung tumorigenesis in the combined group was 30% (6/20), which was also considerably lower than that in the control group 100% (20/20). The incidence of lung tumorigenesis in the shikonin, aconitine and notoginsenoside R1 groups was 95% (19/20), 85% (17/20) and 90% (18/20), respectively, and did not differ significantly in mean tumor size from that in the control group (*p*>0.05), indicating that the used dose of three compounds did not decrease tumor proliferation.

**Fig 2:** The screened three wound healing agents suppressed lung carcinogenesis and their combination led to optimal preventive efficacy. (A) Three wound healing agents were administered to animals following the first carcinogen treatment and were found to prevent lung carcinogenesis. (B) They were administered following the last carcinogen treatment but did not prevent lung carcinogenesis, whereas the combination of these three agents remained effective. (C) Summary data of lung tumor incidence (n = 20). (D) Three wound healing agents restored the lung barrier in urethane-induced lung carcinogenesis. The results are presented as mean±SE (n = 10/group). *p < 0.05, **p < 0.01, vs control group.

**Fig 3:** The screened three wound healing agents desereased lung tumor overall volume and did not negatively impact health or significantly affect the body weights of mice. (A) Three wound healing agents desereased lung tumor overall volume. (B-D) Three wound healing agents did not negatively impact health or significantly affect the body weights of mice. The results are presented as mean±SE (n = 10/group). *p < 0.05, **p < 0.01, vs control group.

In addition, we evaluated lung vascular barrier by EB dye which should not cross through vascular barrier under normal conditions. Urethane-induced lung carcinogenesis increased lung concentration of EB which indicated the increased permeability of the lung vascular barrier. Consistent with decreased carcinogenic incidence, the combination treatment restored the lung vascular barrier to normal levels, whereas single compound did not completely restore the lung vascular barrier (Fig 2D), suggesting that the combination of three compounds led to optimal wound healing.

In this study, the three screened compounds did not appear to be toxic, negatively impact health or significantly affect the body weights of mice at the experimental dose alone or in combination (Fig 3B–3D).

### Urethane-induced lung carcinogenesis was associated with lung injury independent of pulmonary inflammation

To observe whether urethane-induced lung carcinogenesis is associated with pulmonary inflammation or lung injury, mice were intratracheally injected with either BLM or LPS. As shown in Fig 4A–4C, the increased levels of MPO and TNF-α were more in LPS-exposed lungs than those in BLM-exposed lungs compared with normal lung control, in contrast, the increased levels of ROS and 8-OHdG were more in BLM-exposed lungs than those in LPS-exposed lungs, indicating that LPS mainly induce pulmonary inflammation and that BLM mainly induce lung injury although both can not be clearly distinguished. In addition, urethane damaged wound healing in skin excision wound model, and the combination of three compounds led to optimal wound healing in this model (Fig 4D).

**Fig 4:** The combination of three wound healing agents improved urethane-damaged wound healing environment. (A) LPS exposure mainly decreased MPO and TNFα, whereas BLM exposure and macrophage depletion mainly promoted ROS and 8-OHdG. (B) Three wound healing agents improved urethane-damaged wound healing environment (n = 5). (C) Macrophage depletion reversed improved wound healing environment by three compounds alone but had a slight effect on combination efficacy (n = 5). (D) Three wound healing agents promoted wound healing in urethane-induced carcinogenic model (n = 10). The results are presented as mean±SE. *p < 0.05, **p < 0.01, vs urethane carcinogenic group.

In this study, the data from a separate experiment showed that LPS-induced pulmonary inflammation did not result in increased lung carcinogenesis, whereas macrophage depletion decreased pulmonary inflammation but promoted lung carcinogenesis. In contrast, bleomycin-induced lung injury increased lung carcinogenesis. Importantly, all of three conditions decreased carcinogenic preventive efficacy of the single compound but had little effect on combined efficacy (Fig 5A–5D and Fig 6A). The reversed lung carcinogenic efficacy by combination of three compounds was consistent with skin wound healing, and the injured lungs of non-tumor-bearing mice that were treated with the three drugs alone or in combination had returned to normal and showed complete wound healing at terminal sacrifice (S4 Fig), indicating that the carcinogenic preventive efficacy of three compounds could be derived from restoration of a wound healing-like microenvironment.

**Fig 5:** Urethane-induced lung carcinogenesis was associated with lung injury independent of pulmonary inflammation. (A) Urethane-induced lung carcinogenesis was promoted by BLM- or macrophage depletion-induced lung injury but was not affected by LPS-induced pulmonary inflammation. (B-D) LPS exposure, BLM exposure and macrophage depletion reversed carcinogenic preventive efficacy of single compound but had slight effect on combined efficacy shown as lung tumor incidence, lung tumor number and lung weight, respectively. The results are presented as mean±SE (n = 20/group). *p < 0.05, **p < 0.01, vs control group.

**Fig 6:** The combined models increased lung tumor overall volume but did not negatively impact health or significantly affect the body weights of mice. (A) The combined models increased lung tumor overall volume and decreased carcinogenic preventive efficacy of a single compound. (B-E) The combined models did not negatively impact health or significantly affect the body weights of mice. The results are presented as mean±SE (n = 20/group). **p < 0.01, vs control group.

In this study, the combined models or the three screened compounds did not appear to be toxic, negatively impact health or significantly affect the body weights of mice at the end of the experiments (Fig 6B–6E).

### The wound healing-like microenvironment induced by the combination of three compounds decreased lung cancer stem cells

Because cancer stem cells (CSCs) that express stem cell markers are believed to be responsible for the development and progression of many tumors [17], we evaluated the correlation between CSCs and lung tumorigenesis using several putative stem cell markers, including Nanog, Oct4, N-cadherin and vimentin. We also evaluated the expression of normal epithelial E-cadherin and connexin 43 via western blot analysis. The results revealed that carcinogenetic lung tissues expressed more Nanog, Oct4, N-cadherin and vimentin than normal lungs. Conversely, the expression levels of normal epithelial E-cadherin and connexin 43 were decreased. However, treatment with the screened compounds after carcinogen administration decreased the levels of stem cell markers and increased the levels of E-cadherin and connexin 43 to suppress tumorigenesis (Fig 7A and S3 Fig).

**Fig 7:** The wound healing microenvironment decreased lung CSCs and induced cell apoptosis. (A) The combination of three compounds reduced several putative stem cell markers and restored normal E-cadherin and connexin 43 expression examined by western blot analysis in urethane-induced lung carcinogenesis. **(**B) The combination of three compounds decreased expression of the proliferative marker Ki-67 and increased expression of the apoptotic marker cleaved caspase-3 examined by immunohistochemical assays in urethane-induced lung carcinogenesis. The results are presented as mean±SE (n = 5/group) **p < 0.01 *vs* control group. The immunohistochemical images were taken at ×40 magnification.

The ability to proliferate and escape apoptosis is a fundamental property of CSCs. To confirm the presence of CSCs during lung tumorigenesis, immunohistochemical assays using Ki-67 as a proliferative marker and cleaved caspase-3 as an apoptotic marker were conducted with paraffin-embedded lung tissue slides. Ki-67 staining was increased more than 5-fold in carcinogenetic lung tissues compared with normal lungs. Simultaneously, the area that stained positive for cleaved caspase-3 was lower than 20% of the area observed in normal lungs. Furthermore, treatment with the screened compounds alone or combination decreased Ki-67 staining and increased cleaved caspase-3 staining after carcinogen-induced tumorigenesis was suppressed (Fig 7B).

### The wound healing microenvironment induced by the combination of three compounds promoted lung cancer cell differentiation

Dedifferentiation is a fundamental characteristic of tumor cells, especially CSCs [18]. To further study the effect of the wound healing microenvironment on tumor-initiating cells, we treated A549 cells in vitro with the combined compounds as described above. The flow cytometry results showed that the percentage of the population expressing stem cell markers including CD133, Oct4 and Nanog, and EMT markers including N-cadherin, vimentin and snail, greatly decreased in response to treatment with aconitine, especially for the combination of three compounds. However, the effect was not observed for treatment with shikonin or notoginsenoside R1. Simultaneously, exposure to aconitine or the combination of three compounds increased the population that expressed E-cadherin, a normal epithelial marker (Fig 8A).

**Fig 8:** The wound healing microenvironment prevented lung cell malignant transformation. (A) The combination of three compounds reduced the population expressing stem cell markers or EMT markers examined by flow cytometry and in A549 cells. (B) The combination of three compounds decreased A549 cell self-renew shown as the number of tumor spheres and soft agar colonies. (C) The combination of three compounds decreased the population expressing EMT markers examined by flow cytometry in urethane-treated BEAS-2B cells. The results are presented as mean±SE (n = 5/group) **p < 0.01 *vs* control group.

Differentiated cells are characterized by a decreased capacity for self-renewal. To confirm that a wound healing microenvironment can induce differentiation, we carried out tumor sphere formation and soft agar colony formation assays. Consistent with the above results, A549 cells exposed to chronic aconitine or combination of three compounds formed fewer tumor spheres and soft agar colonies than those exposed to control medium. Treatment with other compounds did not affect the number of tumor spheres and colonies compared with control cells (Fig 8B).

### The wound healing microenvironment induced by the combination of three compounds prevented lung cell malignant transformation

The promotion of EMT and loss of GJIC are important characteristics of cell malignant transformation. To support the chemopreventive effect of the wound healing microenvironment on carcinogenesis, we treated BEAS-2B cells in vitro with three compounds alone or in combination to observe urethane-induced cell malignant transformation. Flow cytometric analysis showed a decrease in the population of BEAS-2B cells expressing N-cadherin, vimentin and fibronectin in response to aconitine or combination of three compounds, but the effect was not observed for cells treated with shikonin or notoginsenoside R1. Simultaneously, approximately 10% to 45% of shikonin-treated BEAS-2B cells or BEAS-2B cells treated with the combination of three compounds were E-cadherin-positive cells, whereas less than 10% of urethane-treated cells were E-cadherin positive (Fig 8C).

In contrast, urethane-treated control cells lost GJIC, whereas GJIC was markedly restored in BEAS-2B cells treated with the combination of three compounds; this effect was not observed in shikonin- or aconitine -treated cells (Fig 9A).

**Fig 9:** The wound healing microenvironment restored GJIC but did not directly decrease tumor cells. **(**A) The combination of three compounds reversed GJIC loss in urethane-treated BEAS-2B cells. Images were taken at ×10 magnification. (B and C) The combination of three compounds led to angiogenesis and optimal fibroblast proliferation but did not directly decrease A549 cancer cells. The results are presented as mean±SE (n = 5/group) **p < 0.01 *vs* control group.

To confirm that cancer preventive efficiency was from restoration of a wound healing-like microenvironment but not direct anti-tumor proterties, we treated A549, L929 and ECV304 cells with three compounds alone or in combination. A549 cells were not affected by the used dose of three compounds alone or in combination (more than in vivo plasma concentration). L929 cells were decreased by notoginsenoside R1, not affected by shikonin but were promoted by aconotine and combination of three compounds. ECV304 cells were decreased by shikonin, not affected by aconotine but were promoted by notoginsenoside R1 and the combination of three compounds (Fig 9B and 9C).

## Discussion

The naphthoquinone shikonin is is the major active principle of Lithospermi Radix which is an effective traditional Chinese herb in various types of wound-healing [19]. The combination of shikonin's anti-inflammatory activity together with its wound-healing properties makes it a great potential therapeutic agent for the injury treatment [20], pharmaceutical formulations with wound-healing properties based on shikonin have been in the market for many years although its mechanism of action remains unknown [21].The saponin notoginsenoside R1 (NR1) is the major bioactive component in panax notoginseng which is widely used in Asian countries in the treatment of microcirculatory diseases [22]. The pro-angiogenic action of NR1 in vivo and in vitro provided scientific evidence to be used for the treatment of cardiovascular diseases, traumatic injuries and wound-healing [23]. Aconitine is a major bioactive diterpenoid alkaloid with high content derived from herbal aconitum plants which is widely used to treat various diseases, such as shock caused by acute myocardial infarction, coronary heart disease and angina pectoris in China for thousands of years [24]. However, little information is available on the role of aconitine in wound healing. It was reported that Baikal aconite alkaloids showed manifest wound healing effects on the excision skin wound model [25]. It may be a mechanism of reparative activity to direct stimulation of fibroblasts by aconitine. In our study, although three compounds used alone could promote wound healing, all of them also had unfavorable efficiency to exert wound healing, such as shikonin exerted anti-inflammatory efficiency but decreased angiogenesis and macrophage phagocytosis which was disadvantage in oxygen supply and waste elimination, notoginsenoside R1 stimulated angiogenesis but decreased fibroblasts which was disadvantage in wound healing, and aconitine promoted oxygen supply but intensely stimulated fibroblasts which was unfavorable for correct repair process. The combination of three compounds made up treatment disadvantage of single compound in wound healing and obtained optimal wound healing. Although three compounds have demonstrated their ability to suppress cancer cell proliferation [26–28], the used dose of three compounds alone or in combination had no effect on tumor growth indicated by tumor size in this study. We did not also observe decreased cancer cell proliferation by three compounds alone or in combination in vitro.

One of the core questions in cancer biology relates to the identity and nature of the cancer cell of origin leading to tumor initiation [29]. Evidence from mouse skin models of carcinogenesis suggests that initiated cells at different stages within a stem cell hierarchy require varying degrees of reprogramming depending on their degree of differentiation [30]. For tumorigenesis, various interrelated determinants govern this complex tumor-host interaction, including GJIC, which plays a central role in coordinating intercellular signal-transduction pathways to control tissue homeostasis [31]. In addition, EMT in response to carcinogen exposure supports the involvement of GJIC in the carcinogenesis process [32]. In this study, the wound healing microenvironment decreased the number of lung CSCs, as evidenced by decreased stem cell markers and cell proliferation as well as increased expression of epithelial markers and cell apoptosis. This environment also induced lung cancer cell differentiation, as evidenced by decreased stem cell markers and a capacity of self-renewal, prevented lung cell malignant transformation, as evidenced by decreased EMT and increased GJIC, and delayed tumor progression, as evidenced by the halted progression of hyperplasia to carcinoma in situ or invasive tumors. Our results provide clear evidence that tumor initiation is necessary but not sufficient for tumor formation, and a wound healing microenvironment may induce terminal differentiation, which may in turn cause tumor initiating cells to lose their self-renewal ability and allow their malignant potential to be controlled.

The previous models of chronic wound-associated cancer were usually based on chronic inflammatory microenvironment where regenerative proliferation places the dividing cells at greater risks for acquiring mutations and subsequently selects for those cells that incurred mutations that impart proliferative and/or survival advantages to the cells [33]. Although chronic inflammatory conditions increase cancer risk [34], the hypothesis that the anti-inflammatory activities of celecoxib and aspirin would reduce mouse lung tumorigenesis was not supported in urethane-induced lung carcinogenic model [35]. In this study, we used the mouse-urethane model which exhibits similar histological appearance and molecular changes to human lung adenocarcinoma to evaluate the efficacies of wound healing microenvironment for limitted single agent-elicited carcinogenesis and two-stage carcinogenesis. We found that urethane caused lung injury independent on pulmonary inflammation, and that LPS-induced pulmonary inflammation did not result in increased lung carcinogenesis. In contrast, macrophage depletion decreased pulmonary inflammation but promoted lung carcinogenesis. As expected, bleomycin-induced lung injury increased lung carcinogenesis and the injury increased lung carcinogenesis could be reversed by combination of three compounds but not single compound. In addition, urethane damaged wound healing in skin excision wound model, reversed lung carcinogenic efficiency by the combination of three compounds was consistent with skin wound healing, indicating that the carcinogenic preventive efficacy of three compounds could be derived from restoration of a wound healing-like microenvironment.

In summary, our results suggested that restoration of a wound healing microenvironment represents a simple and effective strategy for cancer prevention. Furthermore, a deficiency in wound healing may be a sensitive index for cancer prognosis.

## Supporting Information

S1 Fig Compound structural formula. (TIF)

S2 Fig Urethane-induced lung histological alteration (× 20). (TIF)

S3 Fig Weastern blot. (TIF)

S4 Fig Wound healing agents restore lung histological structure in urethane-treated mice without lung tumor. (TIF)

S1 Table The screened wound healing agents in mouse skin excision wound model. (TIF)
